# Association of human disturbance and gastrointestinal parasite infection of yellow baboons in western Tanzania

**DOI:** 10.1371/journal.pone.0262481

**Published:** 2022-01-12

**Authors:** Bethan Mason, Alex K. Piel, David Modrý, Klára J. Petrželková, Fiona A. Stewart, Barbora Pafčo

**Affiliations:** 1 Department of Botany and Zoology, Faculty of Science, Masaryk University, Brno, Czech Republic; 2 Institute of Vertebrate Biology, Czech Academy of Sciences, Brno, Czech Republic; 3 Department of Anthropology, University College London, London, United Kingdom; 4 Greater Mahale Ecosystem Research and Conservation (GMERC) Project, Busongola, Tanzania; 5 Institute of Parasitology, Biology Centre, Czech Academy of Sciences, České Budějovice, Czech Republic; 6 Department of Veterinary Sciences, Faculty of Agrobiology, Food and Natural Resources/CINeZ, Czech University of Life Sciences, Prague, Czech Republic; 7 School of Biological and Environmental Sciences, Liverpool John Moores University, Liverpool, United Kingdom; Universidad de Guadalajara, MEXICO

## Abstract

Human disturbance is an ongoing threat to many wildlife species, manifesting as habitat destruction, resource overuse, or increased disease exposure, among others. With increasing human: non-human primate (NHP) encounters, NHPs are increasingly susceptible to human-introduced diseases, including those with parasitic origins. As such, epidemiology of parasitic disease is becoming an important consideration for NHP conservation strategies. To investigate the relationship between parasite infections and human disturbance we studied yellow baboons (*Papio cynocephalus*) living outside of national park boundaries in western Tanzania, collecting 135 fresh faecal samples from nine troops occupying areas with varying levels of human disturbance. We fixed all samples in 10% formalin and later evaluated parasite prevalence and abundance (of isotrichid ciliates and Strongylida). We identified seven protozoan and four helminth taxa. Taxa showed varied relationships with human disturbance, baboon troop size and host age. In four taxa, we found a positive association between prevalence and troop size. We also report a trend towards higher parasite prevalence of two taxa in less disturbed areas. To the contrary, high levels of human disturbance predicted increased abundance of isotrichid ciliates, although no relationship was found between disturbance and Strongylida abundance. Our results provide mixed evidence that human disturbance is associated with NHP parasite infections, highlighting the need to consider monitoring parasite infections when developing NHP conservation strategies.

## Introduction

Parasites can harm host species through a variety of ways, from altering social behaviours [1] to diminishing host physical health and consequently reducing reproductive and foraging success [2]. Parasite infection can further cause damage to neural tissue, reduce fitness, and can even prompt population decline [1, 3], with some infections being fatal to their host [4, 5]. Despite this, parasitic infections in wild animals are often asymptomatic [6, 7], with many hosts coevolving with their parasites overtime [8] and some now believed to be commensals or even mutualists that benefit host physiological functioning, such as aiding digestion [9, 10]. The capacity of parasites to be detrimental to host health may be exacerbated in wild animals that live in fragmented populations or in close contact to human settlements [11], through either increased occurrence of clinical infections [12] or loss of symbiont diversity [10]. This highlights the need to consider the association between human disturbance and parasite infections in wild animals.

Human disturbance has the potential to influence parasite infection of wildlife hosts through multiple indirect mechanisms, such as inducing chronic stress through increased human (predator) encounter rates, urbanisation and noise pollution [13–15], with cascading effects resulting from immunosuppression [16]. Reduced food availability, resulting from habitat disturbance, increases susceptibility to parasites by compromising host nutrition [17, 18]. Additionally, human disturbance may influence parasite infections of wild hosts through transmission from domestic animals, with ongoing agricultural expansion, driven by growing human food demands [19], increasing wildlife to livestock exposure [20]. Livestock proximity has been found to correlate with increased parasite infection in a range of species [21]. Humans can also transfer pathogens to wild animals through reliance on common resources, such as water sources, with poor human sanitation heightening this potential [22, 23]. Transmission from humans is even more likely for non-human primates (NHPs) [6, 24], with their close phylogenetic relationship resulting in numerous shared parasite taxa [21]. Expanding human settlements and fragmentation of wildlife habitat increases human:NHP interactions [6], and thus transmission risk, with forest fragmentation previously linked to increased gastrointestinal parasite infections in western chimpanzees (*Pan troglodytes verus*) [25], among others.

While there are many proposed mechanisms of how human disturbance can influence wildlife hosts, mechanisms are typically taxa specific. *Papio* are known to adapt to anthropogenic environments relatively well [26], in part due to being dietary generalists [27, 28], meaning habitat disturbance is unlikely to influence parasite infections through compromised nutritional status in these hosts. However, higher parasite richness in olive baboons (*P*. *anubis*) has previously been linked with their foraging in anthropogenic habitats [29]. Despite being one of the most terrestrial primates, *Papio* still exhibit arboreal behaviours [30], meaning timber extraction may influence host behaviour. Anthropogenically induced behavioural shifts can increase host exposure risk to parasite infections and consequently shift transmission dynamics, with intensity of timber extraction one factor of human disturbance previously associated with nematode prevalence and infection risk (assessed through a specific index) amongst red colobus (*Piliocolobus tephrosceles*) [31]. Additionally, through either chronic stress or shared parasite taxa, human presence may also influence parasitic infections in *Papio*, as found in lion-tailed macaques (*Macaca silenus*), where increased parasite prevalence and species richness were explained by human presence [17].

Aside from human disturbance, other factors can also influence parasite transmission dynamics. Group size is positively associated with parasite infection in some populations [32]. A variety of mechanisms are proposed for this, including increased exposure resulting from higher animal densities [32] as well as resource competition increasing susceptibility to infection [33, 34]. Age is also associated with parasite infections, with exposure risk and susceptibility to infection influenced by both behavioural and physiological differences between juvenile and adult hosts [35].

For the current study, we focused on nine troops of baboons living within the Basanza Forests of the Uvinza district and Tongwe East and West Forest Reserves, in western Tanzania. The gastrointestinal parasites of baboons are widely documented across *Papio* geographic distribution [29, 36–39]. Gastrointestinal parasites of baboons in Gombe and Mahale Mountains National Parks (Tanzania) have previously been described, identifying nine metazoan and one protozoan species [40]. Despite this extensive documentation of *Papio* parasite infections, little research has focused on the potential impact of human disturbance on these infections. Previously, gastrointestinal symbiont richness in yellow baboons (*Papio cynocephalus*) showed no variation between troops inhabiting protected and unprotected forests in central Tanzania [10]. We compare gastrointestinal parasites of yellow baboons occupying habitat along a gradient of human disturbance in western Tanzania. We investigated troops of differing group size, comprised of both juvenile and adult individuals. We hypothesised that habitat disturbance would be associated with higher prevalence of parasite taxa, resulting from increased transmission risk of previously documented human: NHP shared parasites. We also predicted human disturbance to be associated with higher parasite abundance, due to behavioural shifts and human presence increasing parasite exposure and susceptibility, respectively.

## Material and methods

### Study site

We conducted sampling in Tongwe East and West Forest Reserves within the Greater Mahale Ecosystem and Basanza Forests (Uvinza District) within the Masito-Ugalla Ecosystem, western Tanzania. We selected the Issa Valley (-5.5, 30.54) as a low disturbance area and the outskirts of Uvinza (-5.1, 30.39), a town of >10,000 people ca. 50 km from Issa Valley, as a high disturbance area (Fig 1). In total, we surveyed an area 146 km^2^: ca. 45 km^2^ near Issa Valley and ca. 101 km^2^ near Uvinza. Issa valley is characterised by large expanses of miombo woodland, separated by broad valleys with steep slopes, lined with riparian forests and intermittent grasslands [41, 42]. Uvinza hosts a sprawling town, surrounded by a similar habitat mosaic interspersed with small-scale agriculture and logging sites [43]. Average altitude of sample collection was 1515.5 m in Issa Valley and 1051.3 m in Uvinza, with yearly rainfall around 1000 mm in both areas [41, 42]. Temperature ranges from 11 to 35 °C in Issa Valley [41] and from 20 to 30 °C in Uvinza [44].

**Fig 1:** Study area in western Tanzania. Visual mapping of Tongwe Forest Reserve [45] in Western Tanzania, overlayed with GPS log of faecal collections and transect locations for nine yellow baboon troops, generated in QGIS (v 3.8). Group number is indicated by the boxed number adjacent to transect lines.

### Faecal sample collection

We collected all faecal samples between April and May 2018, spanning the transitional period between the wet (November-April) and dry (May-October) seasons, with dry months defined as those with <60 mm of rainfall [42]. We collected 135 faecal samples of baboons from nine troops (Table 1). One troop (group 1) was habituated and we used individual identifications to ensure no individual was repeatedly sampled, for other troops we collected all faecal samples within a 120 min time period, assuming the limited timespan prevented repeated sampling [46]. We estimated group size by counting all visible individuals prior to sampling, assuming the entire group was counted. We collected samples as soon after defecation as possible (when baboons vacated the immediate vicinity) and stored in sealed sampling pots, with only the central faecal matter being collected to avoid environmental contamination [37, 39]. We recorded a GPS location for each sample and assigned baboon age categories based on size of faeces (juvenile <2 cm faecal diameter; adult >2 cm faecal diameter) [47]. For smaller troops (<15 individuals) we sampled at least 80% of individuals and at least 50% in larger troops (>20 individuals), based on a recommended sample size and gastrointestinal parasite prevalence in olive baboons [18, 39]. Within 180 min of initial collection and storage, we mixed each sample and fixed ca. 3 g of faeces with 10% formalin, storing at room temperature before shipment to the University of Veterinary Sciences, Czech Republic, for analyses.

**Table 1:** Sample collection from yellow baboons in western Tanzania.

Sampling Area	Group	Group Size	Samples Collected		
			Total	Adult	Juvenile
**Issa Valley**	1	13	12	10	2
	2	25	19	19	0
(n = 91)	3	37	19	17	2
	4	21	21	18	3
	8	28	20	19	1
**Uvinza District**	5	5	4	4	0
	6	7	7	6	1
(n = 44)	7	12	10	8	2
	9	29	23	19	4
TOTAL		**177**	**135**	**120**	**15**

Number of samples collected from yellow baboons in western Tanzania split by all relevant factors (sampling area, group, and estimated age).

### Assessing human disturbance

Although we selected two localities with presumably low (Issa Valley) and high (Uvinza District) human disturbance, we still evaluated the human impact directly in the areas occupied by the baboon groups at the time of collection. We assessed human disturbance through a general disturbance index adapted from Barelli et al. [48]. We established five northward orientated 2-km long transects for each sampled troop. Transects were spaced 1 km apart, covering a total area of 8 km^2^ per troop (Fig 1). We recorded all evidence of human disturbance within a five-metre strip of transects, including, but not limited to, roads, livestock, honey production and litter (Fig 2). All signs of tree cutting were also recorded, including cut shrubbery, trees, and any machete marks. We generated transect locations systematically from the faecal collection GPS centroid of each troop, which formed the middle point of the central transect (Fig 1). If natural barriers (e.g., rivers) prevented transect access, we walked additional transects between those that were accessible, ensuring we conducted five transects per troop. If a transect could not be finished due to impassable terrain, the distance completed was used to provide a proportional score. We calculated a mean transect score for each troop then pooled groups by disturbance level based on naturally forming categories: low (< 10 signs) or high (> 300 signs) (Fig 3). Overall, the disturbance levels correspond to the locality which baboon troops inhabit. Areas with high human disturbance are within the Uvinza district (troops assigned high-disturbance level), while low disturbance was observed within the Issa Valley area (groups with low-disturbance level). Interestingly, one group (Group 8, see Fig 3) ranged between these two localities and did not fall into these disturbance categories, (79 signs); we assigned this area with medium disturbance levels, testifying to the declining human activities toward the Issa Valley.

**Fig 2:** Human disturbances observed in the Basanza Forests miombo woodland surrounding Uvinza, Tanzania. (a) Crop agriculture; (b) Livestock agriculture; (c) Cutting signs; (d) Constructional timber production; (e) Charcoal production; (f) Vehicle track.

**Fig 3:** Human disturbances observed in the habitat of yellow baboon troops in western Tanzania. Average human disturbance score, calculated through five transects, recorded in the habitat of nine troops of yellow baboons in western Tanzania, with fill colour depicting the type of human disturbances encountered.

### Faecal sample analysis

We used coproscopic diagnostics by light microscope (Olympus CX40) to determine gastrointestinal parasite diversity and abundance (a proxy for infection intensity) [49]. We diluted samples with water and filtered through gauze before halving sediment to re-fix half (up to 10 ml) in 10% formalin and suspend half (up to 50 ml) in sodium chloride solution [50]. We used the suspended solution to quantify strongylid nematode eggs per gram (EPG), using Mini-FLOTAC apparatus (x100 magnification) and recounting formula. We used the re-fixed sediment to evaluate parasite diversity by Sheather’s flotation [51], documenting all parasite taxa, using cyst, trophozoite and egg morphology for identification [6, 52]. We also examined 0.2 ml of the sediment directly for protozoa diversity (x400 magnification) and evaluation of isotrichid ciliate cyst and trophozoite abundance (CPG = ciliates per gram) [53]. We quantified strongylids and isotrichid ciliates because of their possible pathogenic potential [54].

### Statistical analysis

We performed all statistical analyses using the R statistical interface, R v.3.2.2 [55]. We investigated factors influencing parasite infection, with parasite presence/absence and abundance (measured as EPG/CPG) as response variables, using Generalized Linear Mixed Models (GLMMs). We ran GLMMs using Ime4 package [56] with binomial distribution for presence/absence data and negative binomial distribution for abundance data, to account for the aggregated distribution of parasites within-host population. First of all, our aim was to evaluate the impact of human disturbance level (three categories: low in Issa valley, high in Uvinza district and medium in between these two localities) and further impact of group size and age on the presence/absence and/or abundance of yellow baboon parasites, therefore we set these as explanatory variables. Lastly, as the medium disturbance level was represented by only one group, we set the group affinity as a random factor. We ran a separate model for each parasite and log-transformed the abundance data. Finally, we used Tukey post hoc tests to evaluate differences among levels of factorial explanatory variables in case of disturbance level. We did not use parasite richness to test impact of human disturbance, group size or age, as some parasite taxa (e.g., strongylids and spirurids) comprise multiple species, which are indistinguishable as egg/cysts, which limits the credibility of parasite richness.

### Ethics statement

All protocols were approved by The Animal Welfare and Ethics Steering group at Liverpool John Moores University and adhered to the UK Home Office Animals (Scientific Procedures) Act (ASPA). Research was approved by the Tanzania Commission for Science and Technology (COSTECH), permit no. 2017-320-NA-2011-94, and we collected all samples non-invasively, adhering to Tanzania Wildlife Research Institute (TAWIRI) regulations.

## Results

### Parasite taxa

From the 135 samples examined, we found a total of six protozoan taxa and four helminth taxa (Fig 4), with prevalence data shown in Table 2. We identified three protozoa to species level: *Entamoeba coli*, *Iodamoeba buetschlii* and *Chilomastix mesnili*; and two protozoan taxa to genus level: *Blastocystis* and *Entamoeba* spp. We also noted unidentified isotrichid ciliates. *Entamoeba coli* was identified to species based on the presence of at least eight nuclei, whilst identified *Entamoeba* with alternative nuclei numbers were grouped as *Entamoeba* spp. [35, 57]. Isotrichid ciliates (95.56% positive) and *Entamoeba* spp. (91.11% positive) were the most prevalent protozoa. Four samples were negative for all protozoa. We identified the four helminth taxa based on egg presence, two to genus: *Strongyloides* and *Streptopharagus*, and two to order/suborder (because of microscopically indistinguishable eggs): Strongylida (later strongylids) and Spirurida (later spirurids). *Streptopharagus*’ smaller size compared to other spirurids [58] was used for its distinction. Amongst the helminths, strongylids were the most prevalent, confirmed in all collected samples.

**Fig 4:** Photos of parasites found in yellow baboons’ faeces in western Tanzania. Unidentified isotrichid ciliate cysts: (a) with thick outer protective sheath; (b) without additional protective sheath. (c) Unidentified isotrichid ciliate trophozoites. (d) *Entamoeba coli*. (e) *Entamoeba* sp. (lower cyst) and *Blastocystis* sp. (upper cyst). (f) *Iodamoeba buetschlii*. (g) strongylid egg. (h) *Strongyloides* sp. (i) Spirurid egg. (j) *Streptopharagus* sp.

**Table 2:** Prevalence of gastrointestinal parasites of yellow baboons.

	Prevalence (%)			
	Total	Low disturbance	Medium disturbance	High disturbance
	(135)	(71)	(20)	(44)
Isotrichid ciliates	95.56	100.00	100.00	86.36
*Entamoeba coli*	67.41	76.06	55.00	59.09
*Entamoeba* spp.	91.11	97.18	95.00	79.55
*Iodamoeba buetschlii*	70.37	84.51	55.00	54.55
*Blastocystis* sp.	69.63	63.38	95.00	68.18
*Chilomastix mesnili*	6.67	7.04	0.00	9.09
Strongylids	100.00	100.00	100.00	100.00
*Strongyloides* sp.	23.70	32.39	20.00	11.36
Spirurids	22.96	22.54	25.00	22.73
*Streptopharagus* sp.	44.44	33.80	75.00	47.73

Overall prevalence of gastrointestinal parasites of yellow baboons in Issa Valley and Basanza Forests, western Tanzania, as well as prevalence at each of three disturbance levels. Values in parenthesis indicate number of faecal samples examined.

The mean abundance of isotrichid ciliates was 231.5 EPG, SD: 410.6, and of strongylid nematodes 422.5 EPG, SD: 487.2, in all samples.

### Association with human disturbance

Our transects confirmed higher occurrences of human disturbance in baboon habitat surrounding Uvinza than in Issa Valley, with medium levels of disturbance encountered between the two sites (Figs 1 and 3, Group 8). While a variety of different types of human disturbance were observed, the majority were signs of tree cutting, with livestock and footpaths also frequently occurring.

All parasite taxa were found across all three disturbance levels. Prevalence of two protist and one helminth taxa were associated with disturbance level. The prevalence of *E*. *coli* was significantly associated with disturbance level (GLMM: χ = 126553.0, *p* < 0.001), whereby the prevalence was higher in low disturbance areas compared to high (*p* <0.001). Similarly, the prevalence of *I*. *buetschlii* was significantly different according to disturbance level (GLMM: χ = 13.384, *p* = 0.001), due to being higher in low disturbance areas compared to both in medium (*p* = 0.001) and (although not significant) in high (*p* = 0.066) disturbance areas. Significant differences were observed in distribution levels according to prevalence of *Streptopharagus* sp. (GLMM: χ = 10.106, *p* = 0.006). Significantly higher prevalence of *Streptopharagus* sp. was observed in medium disturbance areas compared to low disturbance areas (*p* = 0.011). Prevalence of other parasite taxa was not significantly associated with disturbance level (S1 Table). Increasing disturbance did show a positive association with isotrichid ciliate abundance (GLMM: χ = 15.8, *p* < 0.001; for results of post hoc tests see Fig 5). Though no significant association with strongylid abundance was found (GLMM: χ = 1.433, *p* = 0.488; Fig 5).

**Fig 5:** Parasite abundance in yellow baboons in western Tanzania. Plots are split by human disturbance of habitat area and show two parasite taxa: (a) unidentified isotrichid ciliate; (b) strongylids.

### Impact of group size and age

The prevalence of *I*. *buetschlii*, *E*. *coli*, *Blastocystis* sp., and *Streptopharagus* sp. was positively associated with group size (GLMM: χ = 14.6981, *p* < 0.001; GLMM: χ = 1024.1, *p* < 0.001; GLMM: χ = 6.478, *p* = 0.011; GLMM: χ = 5.084, *p* = 0.024, respectively) (Fig 6). Additionally, juveniles had increased prevalence of *E*. *coli* (66.6% in adults; 73.3% in juveniles; GLMM: χ = 1777.9, *p* < 0.001) and *Strongyloides* sp. (20% in adults; 53.3% in juveniles; GLMM: χ = 7.365, *p* = 0.007). Prevalence of other parasite taxa was not significantly associated with group size or age (S1 Table).

**Fig 6:** Association between yellow baboon group size and parasite prevalence. Association between group size and parasite prevalence of four parasite taxa amongst yellow baboons situated in western Tanzania.

Group size was significantly associated with isotrichid ciliate abundance (GLMM: χ = 6.99, *p* = 0.008), while strongylids abundance was not (GLMM: χ = 0.321, *p* = 0.571). Age showed no association with abundance of either isotrichid ciliates (GLMM: χ = 0.214, *p* = 0.644) or strongylids (GLMM: χ = 0.064, *p* = 0.801).

## Discussion

Western Tanzania is a mosaic of varied land status, from national parks to open areas, with multiple NHP species, including yellow baboons, distributed throughout, including adjacent to human settlements. To assess the relationship between human disturbance and gastrointestinal parasite infection of yellow baboons, we examined faecal samples from baboon troops inhabiting areas with different levels of human disturbance. Some troops ranged in intact forest areas with minimal human activities, while others ranged closer to human settlements, with larger disturbance signatures, including tree felling, cattle grazing and charcoal production; in some cases, individuals were observed crop raiding.

In general, all ten parasite taxa found in this study are widely reported in yellow baboons from elsewhere [36, 37, 39, 40] as well as in closely related olive and chacma (*P*. *ursinus*) baboons [29, 35]. In *Papio*, gastrointestinal ciliates are typically identified as *Balantioides coli*, however, genetic sequencing of microscopically indistinguishable ciliates, obtained from multiple NHP species, suggests numerous species of *Balantioides*-like and *Buxtonella*-like ciliates inhabit NHP gastrointestinal tracts [59]. Therefore, we report *Balantioides*-like ciliates as ‘unidentified isotrichid ciliates’. One noticeable difference was the absence of *Trichuris* in Issa samples, a parasite widely documented in baboons [29, 36–40], though also absent from savannah chimpanzees (*P*. *troglodytes schweinfurthii*) surveyed in the Issa Valley region [41]. As *Trichuris* is a soil-transmitted helminth (STH), the hot and dry conditions of western Tanzania’s dry season may be unsuitable for the *Trichuris* life cycle, with a low probability of survival during the soil living stage [41]. However, other STH (*Strongyloides* and strongylids) were present, despite requiring a moist external environment for transmission [41]. Examination of all sympatric NHPs would be required to determine if *Trichuris* was absent from specific primate taxa or the entire region, only then yielding further explanation.

In addition, while strongylids are commonly reported amongst baboons, our reported 100% prevalence is high compared to previous studies, where prevalence ranged from 5.9% to 75.4% [10, 38, 40].

### Association with human disturbance

Prevalence of some parasite taxa varied with disturbance level, with most showing decreased prevalence with increased habitat disturbance. Gastrointestinal protozoans and metazoans have previously shown richness reduction in association with habitat degradation in other NHPs: black howler monkeys (*Aloutta pigra*) [60] and Udzungwa red colobus (*Procolobus gordonorum*) [10], although these observations were not mirrored in yellow baboons inhabiting the same area [10]. A reduction in either parasite richness or prevalence could be expected if gastrointestinal protozoans and metazoans respond similarly to human disturbance as many of their animal hosts do, with decreasing population size and diversity [10]. Intuitively, if host numbers, range or densities decrease, the same may be expected for their parasites due to reduced transmission rates [60]. Additionally, conversion of natural habitat for human land use often alters environmental conditions, reducing prevalence of parasite taxa with poor resilience to environmental change [60]. Counterintuitively, reduced gastrointestinal parasite diversity, associated with human disturbance, may be of great concern for wildlife hosts, with many gastrointestinal protozoans and metazoans now considered as vital gut symbionts. These gastrointestinal communities are now believed to be important for maintaining host health and fitness, calling for further research and its inclusion in conservation strategies as a method of endangered species health monitoring [10].

Contrasting findings may be explained by some parasite taxa being more susceptible to the environmental pressures of human disturbance. Convolutions may also arise through microscopic methodologies being unable to reveal all taxa to species or genus level, meaning parasite richness is often a combination of species richness and higher-level taxonomic richness. This calls into question the reliability of parasite richness as a measure for evaluating NHP gastrointestinal parasite communities, with some single parasite taxa in fact representing multiple species.

Besides parasite prevalence, we also evaluated the abundance of strongylids and unidentified isotrichid ciliates according to human disturbance, using EPGs and CPGs respectively. It is debated if intensity of parasite infection is linearly correlated with eggs/cysts shed in faeces, due to temporal variation of egg/cyst output [61–63]. However, with various studies identifying a linear relationship between egg output and adult worm burden within the host [64–66], and a lack of data for wild baboons, we assume egg/cyst output still provides a reliable insight into parasitic infections, as done previously in parasitic research of both *Papio* [39] and other NHP hosts [67–70].

Strongylid nematodes showed no association with level of human disturbance, however, increasing abundances of isotrichid ciliates significantly associated with increased human disturbance. While parasite abundances are less well documented than prevalence data, previous research has shown increases in abundance of other parasite taxa (*Strongyloides* and *E*.*histolytica*) with increases in human disturbance [17, 71]. Human disturbance could potentially increase parasite abundance indirectly through increased chronic stress, with high cortisol (‘the stress hormone’) levels previously correlated with increased parasite susceptibility in NHPs [18]. Alternatively, previous research found *B*. *coli* (an isotrichid ciliate) abundance was higher amongst crop-raiding baboons than wild foraging baboons [29]. While no systematic dietary observations were made here, all troops in the high disturbance area were within one kilometre of cropland and some were seen crop-raiding. Those in the low disturbance area were not in any proximity to cropland. Individuals observed crop raiding were consuming cassava, a highly starch rich crop [72]. Diets high in starch based carbohydrates have been shown to increase *B*. *coli* growth within hosts [73], therefore the increased abundance of isotrichid ciliates in the high disturbance area might be explained by starch rich diets resulting from crop-raiding. While habitat disturbance, due to decreased resource availability, may reduce host nutritional status and thus increase parasite susceptibility in some NHPs [74], this is unlikely to be the case in baboons. *Papio* are typically described as dietary generalists [75], showing adaptability of foraging techniques to anthropogenic food sources [76]. As such, foraging in disturbed areas may in fact be energetically beneficial to *Papio* hosts [77], with anthropogenic food, such as crops, providing nutrient and energy-rich dietary supplementation [60], highlighting the potential impact of increased starch intake as previously mentioned.

### Impact of age and group size

We found group size to be associated with prevalence of some parasite taxa, mostly protozoans, which results from increased animal density and exposure risk amongst larger groups [78]. While sociality, the tendency to form social living groups, has many benefits for wild NHPs [79], increased risk of parasite infection is one well-documented cost [80, 81], with spatial cohesion and contact between individual hosts facilitating parasite transmission [82, 83]. Larger group size may also be associated with higher parasite prevalence due to increased resource competition between group members and social stress amongst host individuals [33, 84] leading to poor nutrition and thus increased parasite susceptibility.

While we found no relationship between age and parasite abundance, we found baboon age to be associated with prevalence of two parasite taxa (*Strongyloides* sp. and *E*. *coli*). Age has previously been linked to parasite prevalence, abundance, and richness in baboons [35, 39], although the direction of these relationships varies between parasite taxa. Increased prevalence in juveniles, as we observed, may be explained by increased susceptibility to parasite infection, less active parasite avoidance or increased exposure risk resulting from age based behavioural differences [35]. Additionally, juveniles may lack fully developed immune systems [85], increasing their susceptibility to parasites [86], while older individuals may acquire immunity to certain parasite stages through repeated exposure [87].

### Conservation implications

Some parasite taxa (*Strongyloides*, *Blastocystis*, *Entamoeba*, isotrichid ciliates and strongylids) found in our samples could have zoonotic potential. However, we highlight that we did not examine inter-specific parasite transmission in this study. *Balantioides coli*, an isotrichid ciliate, is both non-typical and often asymptomatic in humans, though reported in rural areas of some countries [88]. In some cases, *B*. *coli* infection of humans results in diarrhoea with potential for colonic invasion, while rare cases report more serious effects of inflammatory infections and pulmonary haemorrhage [88]. Likewise, *Strongyloides* is also reported in humans and can be asymptomatic [89]. Mixed infections, of multiple *Strongyloides* species, have been reported in both humans and NHPs [25, 90], suggesting zoonotic potential. *Blastocystis* is believed to have larger zoonotic potential, resulting from low host specificity [91]. While *Blastocystis* is commonly reported as part of a healthy human gastrointestinal biome [92], it is also linked to diarrhoea, vomiting and bloating [93]. While *Entamoeba* infection reported in humans is typically of different species to those reported in NHPs, human:NHP shared species have been identified, flagging the zoonotic potential of *Entamoeba* [94]. The symptoms of *Entamoeba* infection are again varied but can cause amebiasis, a potentially fatal intestinal illness [95]. The zoonotic potential of the other parasite taxa found during this study is less understood, although there is still potential for human:NHP transmission [96]. Consequently, shifting patterns of zoonotic parasite infections in wild hosts, resulting from human disturbance, could have implications also for the epidemiology of human parasite infections, heightening the value of considering parasitology within endangered species management.

## Conclusions

Yellow baboons of the Tongwe Forest Reserve exhibit parasite fauna similar to other baboons across Tanzania. Factors influencing both parasite prevalence and abundance varied amongst parasite taxa, providing insight into the complexity of a host’s parasite fauna.

Although we hypothesized that parasite prevalence would increase with human disturbance level, we found the opposite trend, with some taxa showing reduced prevalence in the highly disturbed area. This may result from symbiont organisms showing similar responses to habitat disturbance and degradation as many host species. On the other hand, high levels of human disturbance predicted increased isotrichid ciliate abundance, potentially explained by starch rich diets of baboons in the disturbed area. In future, inclusion of nutritional ecology assays would determine dietary shifts [97] associated with human disturbance, potentially linking with changes in gastrointestinal communities. While measurement of glucocorticoids in faecal samples could provide valuable insight into host stress and fitness [98] and attempt to explain how human disturbance may cause observed differences in gastrointestinal parasite communities.

Further research focused on parasite epidemiology and human:NHP transmission, including sampling of humans and livestock inhabiting the same environment, would be useful in determining the zoonotic parasite risk ongoing habitat disturbance poses to humans. In addition, gastrointestinal communities should be considered as a health monitoring method within NHP conservation strategies, particularly when addressing the threat of human disturbance.

## Supporting information

S1 Table Association of age, group size and habitat disturbance with parasite prevalence. Table showing all statistical results assessing the association between gastrointestinal parasite prevalence in yellow baboons and estimated age, group size and level of habitat disturbance.
(XLSX)

S2 Table Gastrointestinal parasite infections of yellow baboons in western Tanzania. Table showing raw data on gastrointestinal parasite infections of 135 individuals, assessed through coproscopic analysis of faecal samples.
(XLSX)

S3 Table Human disturbance scores of yellow baboon habitat in western Tanzania. Table showing transect scores of transects assessing the human disturbance of natural habitat within the home range of nine yellow baboon troops in western Tanzania.
(XLSX)
